# Multilevel Strip Pooling-Based Convolutional Neural Network for the Classification of Carotid Plaque Echogenicity

**DOI:** 10.1155/2021/3425893

**Published:** 2021-08-18

**Authors:** Wei Ma, Xinyao Cheng, Xiangyang Xu, Furong Wang, Ran Zhou, Aaron Fenster, Mingyue Ding

**Affiliations:** ^1^Medical Ultrasound Laboratory, Department of Biomedical Engineering, College of Life Science and Technology, Huazhong University of Science and Technology, Wuhan 430074, China; ^2^College of Computer Science, South-Central University for Nationalities, Wuhan 430074, China; ^3^Department of Cardiology, Zhongnan Hospital, Wuhan University, Wuhan 430071, China; ^4^Department of Radiology, Liyuan Hospital, Tongji Medical School, Huazhong University of Science and Technology, Wuhan 430077, China; ^5^Department of Ultrasound Imaging, Liyuan Hospital, Tongji Medical School, Huazhong University of Science and Technology, Wuhan 430077, China; ^6^School of Computer Science, Hubei University of Technology, Wuhan 430068, China; ^7^Imaging Research Laboratories, Robarts Research Institute, Western University, London, Ontario, Canada; ^8^Key Laboratory of Molecular Biophysics of Education Ministry of China, Huazhong University of Science and Technology, Wuhan 430074, China

## Abstract

Carotid plaque echogenicity in ultrasound images has been found to be closely correlated with the risk of stroke in atherosclerotic patients. The automatic and accurate classification of carotid plaque echogenicity is of great significance for clinically estimating the stability of carotid plaques and predicting cardiovascular events. Existing convolutional neural networks (CNNs) can provide an automatic carotid plaque echogenicity classification; however, they require a fixed-size input image, while the carotid plaques are of varying sizes. Although cropping and scaling the input carotid plaque images is promising, it will cause content loss or distortion and hence reduce the classification accuracy. In this study, we redesign the spatial pyramid pooling (SPP) and propose multilevel strip pooling (MSP) for the automatic and accurate classification of carotid plaque echogenicity in the longitudinal section. The proposed MSP module can accept arbitrarily sized carotid plaques as input and capture a long-range informative context to improve the accuracy of classification. In our experiments, we implement an MSP-based CNN by using the visual geometry group (VGG) network as the backbone. A total of 1463 carotid plaques (335 echo-rich plaques, 405 intermediate plaques, and 723 echolucent plaques) were collected from Zhongnan Hospital of Wuhan University. The 5-fold cross-validation results show that the proposed MSP-based VGGNet achieves a sensitivity of 92.1%, specificity of 95.6%, accuracy of 92.1%, and F1-score of 92.1%. These results demonstrate that our approach provides a way to enhance the applicability of CNN by enabling the acceptance of arbitrary input sizes and improving the classification accuracy of carotid plaque echogenicity, which has a great potential for an efficient and objective risk assessment of carotid plaques in the clinic.

## 1. Introduction

Ischaemic heart disease and stroke are the leading causes of mortality and morbidity in upper-middle-income and high-income countries [1]. Most strokes and acute coronary syndromes are caused by the rupture of vulnerable atherosclerotic plaques [2], commonly due to the accumulation of fatty deposits at arterial bends and bifurcations. When carotid plaques rupture, atherothrombotic emboli consisting of clumps of platelet aggregates or plaque fragments may travel into the brain, occluding smaller arteries and resulting in a transient ischaemic attack (TIA) or stroke [3]. Ultrasound (US) imaging is a preferred modality for detecting carotid atherosclerotic plaques due to its advantages of being nonionizing, low cost, and convenient for monitoring plaque regression and progression in response to medical therapy [4, 5]. Recent studies have shown that the echogenicity of carotid plaques is associated with their vulnerability [6, 7]. Echolucent plaques are more vulnerable due to their large lipid cores and thin fibrous caps, while echo-rich plaques are stable because they mainly consist of calcifications and fibrotic tissue [8, 9]. The classification of US carotid plaque echogenicity can provide valuable information regarding vulnerable plaques and their risks of causing cerebrovascular events [10–13]. Thus, it is of great significance to identify the echogenicity of carotid plaques, which may contribute to the risk assessment of carotid plaques and be helpful for the risk prediction of cerebrovascular events. However, due to carotid plaques coupled with US image speckles, the complexities of tissue appearances, and the visual similarities of different carotid plaque echogenicities, it is tedious and operator-dependent for expert observers to identify the echogenicity of carotid plaques, and accurate classification is challenging.

Researchers have made some attempts to classify carotid plaque echogenicity using traditional methods based on one or more handcrafted features to tackle this challenge. Irie et al. showed that the greyscale median (GSM) was a useful and objective metric for the assessment of carotid plaque echogenicity for the prediction of cardiovascular events in diabetic patients [14]. GSM was also used as an important feature for the identification of patients with histologically unstable carotid plaques [15]. Prahl et al. used a semiautomated method to evaluate echogenicity (SAMEE) based on a percentage white (PW) feature metric [16]. In [17], a method that combines texture features and morphological characteristics for the assessment of carotid plaque echogenicity was proposed. In [18], a bimodal gamma distribution was proposed to model the pixel statistics in the greyscale images of carotid plaques; the most discriminative features (MDFs) were extracted from the discrete Frechet distance features (DFDFs) of each carotid plaque based on the statistical model to classify the carotid plaques into three types, and a classification accuracy of 77.5% was achieved. In [19], the integral value obtained by calculating the area under the cumulative probability distribution curve (AUCPDC) was adopted to evaluate carotid plaque echogenicity. The classification accuracy for 125 plaques (43 echo-rich, 35 intermediate, and 47 echolucent plaques) was 78.4%, whereas the GSM was 64.8%. All these methods have shown great potential for carotid plaque classification. However, the classification accuracies of the above methods were not high because they used handcrafted features that cannot fully and accurately reflect the complicated intrinsic features of carotid plaques.

Compared to handcrafted features, conventional convolutional neural networks (CNNs), such as VGGNet [20], GoogLeNet [21], and ResNet [22], have been shown to be powerful tools for automatically extracting intrinsic features from medical images [23–25]. A deep convolutional neural network was trained using 129,450 clinical images of skin disease to classify skin lesions in [26]. A multiorgan CAD system based on CNNs was developed for classifying both thyroid and breast nodules and investigating the impact of this system on the diagnostic efficiency of different preprocessing approaches [27]. A deep residual network was applied to automatically extract features of carotid ultrasound images and identify the carotid plaques in the images [28]. A convolutional neural network was built to automatically extract features from carotid ultrasound images for the identification of different plaque components in [29]. The conventional CNN classification tasks require input images of fixed size (e.g., 224 × 224), which contradicts the varying sizes of carotid plaques. Although it is promising to transform carotid plaques of arbitrary sizes to a uniform size by cropping and scaling, as shown in Figure 1, this will result in geometric distortion or changes in the spatial texture features, which may negatively impact the classification accuracy of the utilized model. Although He et al. [30] proved that spatial pyramid pooling- (SPP-) based CNNs could remove the imposed fixed-size constraint and achieve outstanding accuracy in classification and object detection tasks, the limitation of SPP is that it pools the input feature maps with square windows, which is suitable for symmetrical structure, such as the lumen of the artery. While this limits the flexibility in capturing the anisotropy context that widely exists in carotid plaques, because carotid plaques are mainly formed by an accumulation of lipid and inflammatory deposits in the subintimal space of the arterial wall, during this process, affected by the hemodynamics in the vascular lumen, most of the carotid plaques are long strips in the longitudinal section of carotid ultrasound (e.g., the carotid plaques in Figures 2(e) and 2(f)). The pooling operation using square windows in SPP cannot overcome the aforementioned limitation efficiently because it will inevitably contain information about contamination from irrelevant areas.

To this end, in this study, we considered that most carotid plaques ultrasound images in the longitudinal view are stripe-like structure, and MSP was proposed for the classification of carotid plaques, which pools the feature maps using multilevel stripped shape windows and obtains fixed length outputs, which are then fed into the fully connected layers. MSP not only inherit the merits of SPP, which can accept input images of any size, but also enlarge the receptive field and maximum effectively capture the long-range context in the longitudinal view to improve the accuracy for the classification.

The main contributions of our work can be generalized as follows.

We investigate the design of the SPP module and propose an MSP module, which inherits the advantage of SPP that can accept input images of arbitrary size and overcomes the limitation of SPP to more effectively capture long-range context to improve the classification performance.

Furthermore, we present an MSP-based CNN for the automatic and reliable classification of carotid plaque echogenicity, which achieves significant improvements over the baseline VGG16, SPP-based CNN, and other popular CNNs and enables efficient stability estimations of carotid plaques so that clinicians can make suitable diagnostic schemes.

A large-scale clinical carotid US dataset was established for carotid plaque classification. The dataset includes 1463 carotid plaque US images, which consist of three different carotid plaque types according to their echogenicity. Each carotid plaque in this dataset has a classification label and its corresponding region of interest (ROI).

The remainder of this paper is organized as follows.  Section 2 introduces the preparation of the dataset and the structures of the SPP module, the proposed MSP module, and the MSP-based CNN.  Section 3 describes the experimental setup and utilized classification metrics and presents the experimental results and discussion, and conclusions are given in Section 4.

## 2. Materials and Methods

### 2.1. Data Acquisition and Preparation

#### 2.1.1. Data Acquisition

In this study, a total of 1463 US images of carotid plaques were acquired from 925 patients in Zhongnan Hospital of Wuhan University by expert sonographers who have decades of experience in vascular imaging. An Acuson SC2000 (Siemens, Erlangen, Germany) US system equipped with a 5-12 MHz linear array probe (9L4) was used to acquire carotid US images. This study was approved by the Institutional Review Board (IRB) of the Medical School, Wuhan University, and written informed consent was obtained from all patients. During the acquisition process, the subjects were supine, and their heads were tilted back. The probe was positioned perpendicular to each patient's neck, moving slowly along the carotid arteries. After a carotid plaque was identified, longitudinal images of the carotid plaque in the common and internal carotid arteries were acquired.

#### 2.1.2. Data Preparation

*(1) Image Normalization*. The appearances of carotid US images vary due to different image acquisitions depending on the equipment, operator, patient, and US machine settings. Consequently, it is important to develop methods that can address the variability in the appearances of tissues in US images. Traditionally, image normalization is used to overcome this limitation, i.e., by transforming the image data such that the same tissues have approximately similar intensity values. In this paper, the proposed deep learning network can extract high-level features from carotid US images; therefore, these features are less sensitive to image normalization. To improve the comparability of the images and the reliability of our results, we applied a linear scaling operation between the minimum and maximum values of the images as a standard processing method for normalization (without the need for any user interaction). The normalization formula is defined by (*x* − *x*_min_)/(*x*_max_ − *x*_min_), where *x* is the pixel value of a carotid plaque US image and *x*_min_ and *x*_max_ are the minimum and maximum pixel values of this carotid plaque US image, respectively.

*(2) Groundtruth Data*. Our groundtruth data were generated according to the criteria of the European carotid plaque study group, which classified carotid plaque echogenicity into three different types: echo-rich, intermediate, and echolucent [31]. This classification was performed by an expert clinician (coauthor F.W.) with at least a decade of experience in the assessment of atherosclerosis using carotid US images, who first classified 1463 plaques into three categories based on their echogenicity (echo-rich, intermediate, and echolucent) and reclassified them three months later. The kappa value (*κ* = 0.747) was calculated to demonstrate that the two classifications had high intraobserver agreement. For the 232 controversial plaques, Dr. Wang classified them for a third time and then took two of the three results that were consistent with the final results. Ultimately, the groundtruth data included 335 echo-rich plaques, 405 intermediate plaques, and 723 echolucent plaques among all 1463 plaque images.

*(3) Manual Segmentation of Plaques*. Due to the large sizes of the acquired images and the fact that the area outside each plaque did not contain critical related information, the boundaries of the plaque were manually delineated for each image by the same expert clinician, and then, the ROI containing the segmented plaque was saved, as shown in Figure 1. An automatic segmentation method for carotid plaques is being studied by another member of our laboratory [32]. Because segmentation is not the focus of this study, the manual segmentation results were used as the ROIs. These ROIs containing plaques vary in size, with the largest size being 134 × 564 (*h* × *w*) and the smallest one being only 19 × 29 (*h* × *w*).  Table 1 shows the statistical distribution and sizes of the samples per class for training and testing obtained from one of the conducted 5-fold cross-validation.

### 2.2. Spatial Pyramid Pooling (SPP) Module

Before describing the design of MSP, as depicted in Figure 3, we first briefly review the structure of the SPP module. In this module, the pooling operations are performed with a pyramid level of *a*_*n*_ × *a*_*n*_ bins for the *k* feature maps obtained after the last convolutional layer and a size of *m*_*h*_ × *m*_*w*_. The size of the sliding pooling window is ⌈*m*_*h*_/*a*_*n*_, *m*_*w*_/*a*_*n*_⌉, and the stride is ⌊*m*_*h*_/*a*_*n*_, *m*_*w*_/*a*_*n*_ ⌋, where ⌈·⌉ and ⌊·⌋ denote the ceiling and floor operations. The outputs of the *j*-level pyramid pooling layer can be calculated by *k*∑_*n*=1_^*j*^*a*_*n*_^2^, where *k* is the number of filters in the last convolutional layer, and *a*_*n*_^2^ denotes the bins of level *n* of the pyramid pooling layer. As an example, a 3-level pyramid pooling layer {3 × 3, 2 × 2, 1 × 1} results in 14 bins. Finally, the outputs of the 3-level pyramid pooling layer are concatenated to obtain *k*∑_*n*=1_^3^*a*_*n*_^2^(*a*_1_ = 1, *a*_2_ = 2, *a*_3_ = 3)14*k* fixed-dimensional vectors and input them into the fully connected layer to obtain the classification results.

### 2.3. Multilevel Strip Pooling (MSP) Module

SPP can generate a fixed-length representation that does not depend on the size of the input image. However, it pools the feature maps using square windows to collect context, which would inevitably contain contaminating information from irrelevant regions. This is especially true for long-strip targets such as carotid plaques in the longitudinal section of the carotid ultrasound images. Thus, inspired by [33], we designed a novel MSP module to alleviate the above problem. It uses multilevel strip-shaped window to enlarge the receptive field and perform strip pooling to allow the collection of long-range contexts, as shown in Figure 4.

Let the size of the *k* feature maps obtained from the previous convolution layer be *m*_*ih*_ × *m*_*iw*_(*i* = 1, 2, ⋯*N*) (*N* is the sample size of the dataset). In the *n*th level strip pooling of *a*_*n*_ × *b*_*n*_ strips, we adopt adaptive average pooling with a kernel (*k*_*h*_, *k*_*w*_) and stride (*s*_*h*_, *s*_*w*_) to obtain the output. The kernel (*k*_*h*_, *k*_*w*_) and stride (*s*_*h*_, *s*_*w*_) can be calculated as follows:

(1) $$\begin{array}{c} s_{h}=\left\lfloor \frac{m_{ih}}{a_{n}}\right\rfloor ,\\ k_{h}=m_{ih}-\left(a_{n}-1\right)s_{h},\\ s_{w}=\left\lfloor \frac{m_{iw}}{b_{n}}\right\rfloor ,\\ k_{w}=m_{iw}-\left({\text{b}}_{n}-1\right)s_{w}. \end{array}$$

Then, *j*-level strip pooling operations are performed on each feature map (the response of each filter) using a strip-shaped window in the horizontal or vertical dimension. Similar to those obtained with spatial pyramid pooling, the output vectors *v*_*o*_ after *j-*level strip pooing can be written as

(2) $$\begin{array}{c} v_{o}=k\overset{j}{\underset{n=1}{\sum }}a_{n}\times b_{n}. \end{array}$$

Here, *j* is the number of levels, and *k* denotes the number of filters of the last convolutional layer in the backbone network. Thus, the number of output vectors obtained after the above strip pooling operation is fixed for all feature maps. The MSP layer pools the features and generates fixed-length vectors, which are then fed into the fully connected layers for the classification of carotid plaques. As an example, a 3-level strip pooling layer with strips of {1 × 1, 2 × 1, 3 × 1} in horizontal dimension results in 6 strips. Then, we concatenate the outputs of the 3-level strip pooling layer to obtain *k*∑_*n*=1_^3^*a*_*n*_ × *b*_*n*_(*a*_1_ = 1, *a*_2_ = 2, *a*_3_ = 3; *b*_1_, *b*_2_, *b*_3_ = 1)6*k* fixed-dimensional vectors and input them into the fully connected layer for the classification.

It should be noted that Figure 4 only shows multilevel strip pooling in the horizontal dimension. In fact, each feature map can be pooled by the MSP module using a multilevel strip window to average all the feature values in the horizontal, vertical, or both dimensions. In image classification, we can flexibly choose horizontal, vertical, or both dimensions multilevel strip pooling according to the structural characteristics of the target object in the image. The outputs of the multilevel strip pooling operations are fixed-dimensional vectors, which contain global and local informative contexts. In this study, since we collected carotid plaques in the longitudinal section of carotid US images, the long-range context in the horizontal dimension is more informative. According to the results of the preliminary experiment, to take efficiency into account and to make the MSP module lightweight, in this work, we adopt MSP operations only in the horizontal dimension to capture multilevel long-range context of carotid plaques. For example, in Figure 4, the vector bounded by the red box in the outputs is obtained by pooling the horizontally long-range area (enclosed by the red box) of the feature maps using one of 3 × 1 strips in the 3rd-level strip pooling. Compared to SPP, MSP considers using long but narrow kernel instead of square window for pooling, which focuses on acquiring long-range context in horizontal dimension and avoiding some unnecessary connections to be built in vertical dimension. Furthermore, the module is an add-on building block that can be plugged into the backbone of any network. In the following, we describe the structure of the proposed MSP-based CNN for the classification of carotid plaque echogenicity.

### 2.4. MSP-Based CNN for the Classification of Carotid Plaque Echogenicity

The VGG model is one of the most popular deep learning networks because it reinforces the notion that CNNs must have a deep network of layers for a hierarchical representation of visual data to be possible. Although many follow-up works have improved upon the VGG architecture, in this work, we used the VGG network with a simple structure as the backbone to build the MSP-based CNN.

The structure of MSP-based VGGNet, as shown in Figure 5, consists of two main components. One component employs the same 5 convolution and pooling blocks as VGG16, except for the pooling layer after the last convolution layer, which is mainly used for image feature extraction. Each block has multiple convolution layers (with rectified linear unit (ReLU) activation), which use 3 × 3 filters with strides and paddings of 1, along with 2 × 2 max-pooling layers with strides of 2. The convolution layers operate in a sliding window manner to perform feature extraction on the input carotid plaque images of arbitrary sizes and generate feature maps of any size. The other component is the MSP module, followed by the fully connected layer and Softmax layer. The MSP module can perform multilevel strip pooling on the acquired feature maps of arbitrary sizes to obtain a fixed-size feature representation and then input it into the fully connected layer for carotid plaque echogenicity classification.

To prevent the model from overfitting, we use publicly available weights for the VGG16, trained against the ILSVRC12 challenge dataset and fine-tune them through transfer learning [34] for our purpose. Meanwhile, a dropout layer [35] is added to the network before the last fully connected layer. The feed-forward operation in the network with dropout is shown in Equations (3)–(6). Here, the Bernoulli function will randomly generate a vector of 0 or 1. *z*^*l*^ denotes the vector of inputs into layer l, and *y*^(*l*)^ denotes the vector of outputs from layer *l*. *w*^(*l*)^ and *b*^(*l*)^ are the weights and biases at layer *l* [35].

(3) $$\begin{array}{c} r_{j}^{\left(l\right)}∼\text{Bernoulli}\left(p\right), \end{array}$$

(4) $$\begin{array}{c} {\tilde{y}}^{\left(l\right)}=r^{\left(l\right)}*y^{\left(l\right)}, \end{array}$$

(5) $$\begin{array}{c} z_{i}^{\left(l+1\right)}=w_{i}^{\left(l+1\right)}{\tilde{y}}^{l}+b_{i}^{\left(l+1\right)}, \end{array}$$

(6) $$\begin{array}{c} y_{i}^{\left(l+1\right)}=f\left(z_{i}^{\left(l+1\right)}\right). \end{array}$$

## 3. Results and Discussion

In this section, we implement MSP-based VGGNet for the classification of carotid plaque echogenicity on the collected dataset, which was labelled three types (echo-rich, intermediate, and echolucent).

### 3.1. Experimental Setup

We used an open-source deep learning framework, PyTorch, for training and testing the proposed network and popular CNNs for comparison purposes. All training and testing procedures were performed on an Ubuntu 64-bit desktop personal computer with an Intel Core i9-10900K central processing unit (CPU) and 32 GB of random access memory. An NVIDIA RTX 2080 Ti graphical processing unit (GPU) with CUDA 10.1 was used for acceleration.

The cross-entropy function was used as the cost function, and the stochastic gradient descent (SGD) optimizer was adopted to minimize the cost function [36]. The number of iterations was 30, the momentum was 0.9, and the learning rate was set to 0.001, which was reduced by a factor of 10 after every 6 iterations.

During the training and testing phases, we used batch data to train the network. The batch data needed to be consistent in all dimensions because the batch array was required to be converted into a tensor during the training and testing phases. Consequently, the batch size should be set to 1 when using SPP-based VGGNet and MSP-based VGGNet accepted images with arbitrary sizes as inputs.

### 3.2. Evaluation Metrics

The performances of networks in terms of carotid plaque classification were evaluated using the accuracy, sensitivity (recall), specificity, precision, and F1-score metrics, which are defined as follows:

(7) $$\begin{array}{c} \text{accuracy}=\frac{\text{TP}+\text{TN}}{\text{TP}+\text{FP}+\text{TN}+\text{FN}},\\ \text{sensitivity}=\frac{\text{TP}}{\text{TP}+\text{FN}},\\ \text{specificity}=\frac{\text{TN}}{\text{TN}+\text{FP}},\\ \text{precision}=\frac{\text{TP}}{\text{TP}+\text{FP}},\\ \text{F}1‐\text{score}=\frac{2\times \text{precision}\times \text{recall}}{\text{precision}+\text{recall}}, \end{array}$$

where TP, FP, TN, and FN represent the numbers of true positive, false positive, true negative, and false negative cases, respectively. Sensitivity measures the ability to correctly recognize positive cases, while specificity indicates the ability to correctly classify negative cases. Precision denotes the proportion of positive cases that were classified as positive cases, and the F1-score represents the harmonic average of precision and recall and is typically used for the optimization of a model towards either precision or recall.

### 3.3. Experimental Results

We designed three experiments to investigate the effects of various levels and pools in the SPP and MSP modules and chose the best module to demonstrate the effectiveness of MSP-based VGGNet for the classification of carotid plaque echogenicity by comparing it with the baseline network VGG16 and SPP-based VGGNet, and to compare it with other popular CNNs.

#### 3.3.1. Selection of the Levels and Pools in MSP and SPP Modules

To verify whether the number of levels and pools affects the experimental results, we explored the effect of a 4-level strip pooling layer with strips of {1 × 1, 2 × 1, 3 × 1, 4 × 1}, namely, MSP-1234, and three 3-level strip pooling layers with strips of {1 × 1, 2 × 1, 3 × 1}, {1 × 1, 2 × 1, 4 × 1}, and {2 × 1, 3 × 1, 4 × 1}, namely, MSP-123, MSP-124, and MSP-234, respectively. The settings and outputs are described in Table 2, and the results are presented in Figure 6(a). The accuracy of MSP-123 reached 0.921, which was also slightly higher than that in the other cases. More levels, such as in MSP-1234, or more strips, such as in MSP-124 and MSP-234, provided very little in terms of performance gains. This may be due to sufficient long-range information being collected with MSP-123.

A similar pooling configuration was applied in SPP-based VGGNet. A 4-level SPP layer with a pool of {1 × 1, 2 × 2, 3 × 3, 4 × 4}, namely, SPP-1234, and three 3-level SPP layers with varying pools of {1 × 1, 2 × 2, 3 × 3}, {1 × 1, 2 × 2, 4 × 4}, and {2 × 2, 3 × 3, 4 × 4}, namely, SPP-123, SPP-124, and SPP-234, respectively, were verified in SPP-based VGGNet. The settings used are also shown in Table 2. The results are depicted in Figure 6(b), which shows that the accuracy of SPP-123 was also slightly higher than that in the other cases, especially at the beginning of epochs below 7. There were no significant differences between the accuracies of the other two pools in the 3-level spatial pyramid pooling layer and the 4-level spatial pyramid pooling layer.

As a result, regarding the runtime cost, we adopted a 3-level strip pooling layer with a strip of {1 × 1, 2 × 1, 3 × 1} in MSP-based CNNs, that is, MSP-123 and a 3-level SPP layer with a pool of {1 × 1, 2 × 2, 3 × 3} in SPP-based CNNs, that is, SPP-123 as the default settings in the following experiments.

#### 3.3.2. Effectiveness of MSP-Based VGGNet

We demonstrate the effectiveness of MSP-based VGGNet on the collected dataset for the classification of carotid plaque echogenicity. The 5-fold cross-validation procedure was adapted to obtain more impartial and unbiased results. To evaluate the performance of the proposed MSP-based VGGNet, we compared it with the baseline VGG16 network and SPP-based VGGNet, and the results are shown in Figure 7 and Tables 3 and 4. From Figure 7, it can be seen that the proposed MSP-based VGGNet obtained the highest accuracy, and the testing process was stable and converged quickly.

The performance metrics obtained on our dataset other than accuracy are shown in Tables 3 and 4, where SEN_ER_, SEN_IM_, and SEN_EL_ represent the sensitivities of the networks to the echo-rich plaques, intermediate plaques, and echolucent plaques, respectively, and SPE_ER_, SPE_IM_, SPE_EL_, PRE_ER_, PRE_IM_, PRE_EL_, F1‐score_ER_, F1‐score_IM_, and F1‐score_EL_ denote the respective specificities, precisions, and F1-scores. $\bar{\text{SEN}}$ represents the overall mean classification sensitivity, which combines SEN_ER_, SEN_IM_, and SEN_EL_ for the three different types of plaques, and $\bar{\text{SPE}}$, $\bar{\text{PRE}}$, and $\bar{\text{F}1‐\text{score}}$ represent the corresponding overall mean specificity, precision, and F1-score, respectively.

Tables 3 and 4 show that our proposed MSP-based VGGNet performed better than VGG16 and SPP-based VGGNet in terms of classifying the three types of plaques. On the echo-rich plaques, the mean sensitivities of MSP-based VGGNet according to 5-fold cross-validation were 95.9 ± 2.3%, which surpassed those of VGG16 and SPP-based VGGNet by 17.9% and 1.1%, respectively. The mean specificities, precisions, and F1-scores were also higher than those of VGG16 and SPP-based VGGNet. This finding was also evident for the intermediate plaques. On the echolucent plaques, although VGG16 provided the best mean sensitivity (92.9 ± 2.3%), it had relatively low specificity (79.4 ± 2.8%), precision (82.9 ± 1.8%), and F1-score (87.6 ± 1.7%). By comparison, our MSP-based VGGNet not only provided the second-ranked sensitivity (92.8 ± 2.0%), which was very close to the best sensitivity (92.9 ± 2.3%) with no statistically significant difference between them (*p* = 0.4), but also obtained the best specificity (93.3 ± 2.0%), precision (93.2 ± 1.8%), and F1-score (93.0 ± 1.2%). Moreover, the overall average sensitivity of 92.1 ± 1.3%, specificity of 95.6 ± 0.5%, precision of 92.0 ± 0.5%, and F1-score of 92.1 ± 0.8% obtained by our MSP-based VGGNet are higher than those of VGG16 and SPP-based VGGNet, which also demonstrates the superiority of the proposed method.

Finally, comparisons of the training and testing times of the three tested networks are provided in Table 5. It can be seen that the least time was spent by our MSP-based VGGNet during the training and testing phases due to it having fewer parameters and reduced computational costs.

#### 3.3.3. Classification Comparison with Popular CNNs

Figure 8 shows a comparison of our proposed network with several popular CNNs. Obviously, our MSP-based VGGNet achieved accuracy higher than 0.9, which was much better than those of all the popular networks. Meanwhile, our proposed network converged after almost 5 epochs on the test set, which was faster than other networks, and the training process is more stable. Among the compared popular CNNs, they had similar classification performance. ResNet50 had a slightly higher accuracy, while the latest EfficientNet-b7 had a slightly lower accuracy. This indicates that it is not that the more complex the network architecture is, the better is the classification performance. Our specially designed network had a simpler architecture but should be more suitable for the classification of specific medical images than the complex heavy-weighted networks in the case of a small dataset.

Figure 9 shows the confusion matrices of ResNext50 [37], DRN-d22 [38], MobileNet-v2 [39], DenseNet121 [40], EfficientNet-b7 [41], and MSP-based VGGNet for the classification of the three types of carotid plaques using 5-fold cross-validation. From Figure 9, it is apparent that our proposed network provided the best classification rates for the three types of plaques. All the CNNs achieved similarly high correct classification rates (ranging from 0.903 to 0.927) for the echolucent plaques, but the classification rates of MSP-based VGGNet for the echo-rich and intermediate plaques are significantly higher than those of popular CNNs. Especially for the intermediate carotid plaques that are difficult to distinguish, our proposed network achieves an accuracy of 0.876, while the highest accuracy among popular CNNs is 0.766 obtained by DRN-d22. The accuracy of MobileNet-v2 in this category is lower than 0.700. Although EfficientNet-b7 achieved the second highest recognition rate of 0.852 for echo-rich plaques, it was 10.7% lower than our proposed network. Meanwhile, it performed poorly in the classification of intermediate plaques, which misclassified 30.9% of the intermediate plaques as echolucent plaques, and provided the lowest recognition rate of 0.582 for the intermediate plaques among popular CNNs. Overall, our MSP-based VGGNet provides the best classification results for the classification of carotid plaques echogenicity.

For a comparison with the traditional methods, the GSM and AUCPDC values of all 1463 images were calculated based on the greyscale distribution, and then, they were used by a support vector machine (SVM) classifier to classify the plaques according to the three different types. However, the results obtained were poor and are not shown here.

## 4. Discussion

The accurate and objective classification of carotid plaque echogenicity is crucial for stroke risk assessment and for the planning of optimal treatment strategies. In this study, we proposed MSP-based CNN for the classification of carotid plaque echogenicity, which differs from the previous work. In particular, previous classification methods [16–19] identified different types of carotid plaques using handcrafted features, which lacked the ability to achieve a potential higher performance due to their inability to comprehensively represent the complicated features of carotid plaque. Meanwhile, obtaining these handcrafted features required professional domain knowledge and manual intervention, which limits the applicability of the method for other classification tasks. In contrast, the proposed approach can automatically extract low- and high-level features from the massive carotid plaques and serve the classification purpose without requiring manual intervention, suggesting the utility in research and clinical studies. Compared to the popular CNNs, the proposed MSP-based CNN can accept carotid plaques of arbitrary sizes as inputs, while popular CNNs need to transform the input images to a uniform size by cropping and scaling, which will cause content loss or distortion and hence has a negative impact on the classification accuracy. Although the widely used SPP network can also accept input images of any size, its ability to exploit anisotropy contextual information is limited since only square kernel shapes are applied. In contrast, our MSP-based CNN has a couple of advantages. First, it enlarges the receptive field by strip pooling and has less network parameters that resulted in less computational cost. Secondly, considering that the ultrasound images of carotid plaques in the longitudinal section are generally stripe-like structure and the greyscale distribution is anisotropic, the proposed MSP-based CNN adopts multilevel strip pooling in horizontal dimension to capture more accurate context, which is beneficial to improve the classification accuracy of carotid plaques. Experimental results show that the proposed MSP-based CNN is superior in terms of discriminating the three different types of carotid plaques compared to popular CNNs and SPP-based CNN.

Although we achieved high classification accuracy as well as computational efficiency, we must acknowledge a number of limitations. We note that the recognition rate of intermediate plaques is lower than echo-rich and echolucent plaques. This may be because of the complex morphology and variability of intermediate plaques. We may consider the novel attention mechanism to more accurately capture the information closely related to the classification task, while eliminating some irrelevant information, so as to improve the recognition rate. In addition, the groundtruth for this study was provided by only one expert clinician with decades of experience working with carotid ultrasound data. In the follow-up study, the generation of groundtruth datasets by multiple experts from different institutions would be needed to evaluate the sensitivities of the proposed networks on the training dataset and ensure that the results are generalizable. Furthermore, patients should be followed for at least 5 years and their carotid plaques should be reclassified to determine if the plaques are changing and becoming unstable, and patient outcome data (i.e., TIAs or strokes) should be compared to the classification results to determine if these data can be used clinically as risk indicators.

## 5. Conclusions

In this work, we investigated the design of the SPP module, proposed the MSP module, and presented MSP-based VGGNet to improve the classification performance with respect to carotid plaque echogenicity. A 5-fold cross-validation was used to evaluate the effectiveness of our network on a collected clinical dataset. In a comparison with popular CNNs, the experimental results demonstrated that our network is more effective for correctly classifying the echogenicity of carotid plaques into three types. Therefore, our network may potentially assist clinicians in using a more objective risk assessment metric for carotid plaques to monitor plaque changes and predict possible cerebrovascular events.

## Figures and Tables

**Figure 1:** A plaque with a size of 49 × 234 was transformed to a uniform size of 224∗224.

**Figure 2:** Three examples of manually segmented carotid plaques. (a–c) Three US images of three types of plaques: echo-rich, intermediate, and echolucent, respectively. (d–f) Images of the plaques that were manually segmented by an experienced clinician. (g–i) The ROIs that contain the plaques.

**Figure 3:** The structure of SPP module. Here, *k* is the number of feature maps.

**Figure 4:** The structure of MSP module. Here, *k* is the number of feature maps.

**Figure 5:** The structure of MSP-based VGGNet. Here, the number of filters in the last convolutional layer is 512.

**Figure 6:** The effects of various levels and pools on classification accuracy.

**Figure 7:** Accuracy comparison among MSP-based VGGNet, SPP-based VGGNet, and VGG16.

**Figure 8:** Accuracy comparison with popular networks in terms of carotid plaque classification.

**Figure 9:** Confusion matrices of the compared networks for the classification of carotid plaques. ER, IM, and EL represent echo-rich plaques, intermediate plaques, and echolucent plaques, respectively.

**Table 1:** Statistics distribution and sizes of our collected dataset.

Types of plaques	Images	Training set	MaxSize	MinSize	Testing set	MaxSize	MinSize
Echo-rich	335	266	99 × 259	19 × 29	69	84 × 285	28 × 44
Intermediate	405	315	134 × 564	37 × 67	90	129 × 549	40 × 108
Echolucent	723	588	93 × 569	29 × 69	135	116 × 563	27 × 87
Total	1463	1169	134 × 564	19 × 29	294	129 × 549	28 × 44

**Table 2:** Different settings and outputs in MSP and SPP.

Name	Level				Total strips/bins	Outputs
	1^st^	2^nd^	3^rd^	4^th^		
MSP-123	1 × 1	2 × 1	3 × 1	—	6 strips	6*k*
MSP-124	1 × 1	2 × 1	4 × 1	—	7 strips	7*k*
MSP-234	2 × 1	3 × 1	4 × 1	—	9 strips	9*k*
MSP-1234	1 × 1	2 × 1	3 × 1	4 × 1	10 strips	10*k*
SPP-123	1 × 1	2 × 2	3 × 3	—	14 bins	14*k*
SPP-124	1 × 1	2 × 2	4 × 4	—	21 bins	21*k*
SPP-234	2 × 2	3 × 3	4 × 4	—	29 bins	29*k*
SPP-1234	1 × 1	2 × 2	3 × 3	4 × 4	30 bins	30*k*

**Table 3:** Sensitivity and specificity comparisons among VGG16, SPP-based VGGNet, and MSP-based VGGNet.

Fold	Methods	Performance evaluation (%)							
		SEN_ER_	SEN_IM_	SEN_EL_	$\bar{\text{SEN}}$	SPE_ER_	SPE_IM_	SPE_EL_	$\bar{\text{SPE}}$
1	VGG16	82.6	73.3	**92.6**	82.8	96.5	92.9	83.1	90.8
	SPP-VGG	95.7	91.1	87.4	91.4	97.6	92.5	94.9	95.0
	MSP-VGG	**98.6**	**91.1**	89.6	**93.1**	**98.1**	**94.5**	**94.9**	**95.8**

2	VGG16	84.6	67.5	92.8	81.6	98.0	91.2	82.3	90.5
	SPP-VGG	98.5	87.0	**93.4**	93.0	97.7	**96.3**	94.3	96.1
	MSP-VGG	**98.5**	**90.9**	92.8	**94.1**	**98.1**	95.8	**95.7**	**96.6**

3	VGG16	70.8	66.7	**94.3**	77.3	98.9	88.5	77.8	88.4
	SPP-VGG	91.7	76.5	90.1	86.1	97.9	92.8	86.5	92.4
	MSP-VGG	**94.4**	**85.2**	92.9	**90.9**	**99.5**	**94.8**	**90.7**	**95.0**

4	VGG16	78.8	64.9	96.0	79.9	**99.0**	92.9	77.3	89.7
	SPP-VGG	93.9	81.8	96.0	90.6	97.6	**97.2**	90.6	95.1
	MSP-VGG	**95.5**	**81.8**	**96.0**	**91.1**	98.6	96.3	**91.3**	**95.4**

5	VGG16	73.1	63.4	89.0	75.2	**99.5**	84.8	76.5	86.9
	SPP-VGG	**94.0**	85.4	89.0	89.5	97.6	92.8	91.7	94.0
	MSP-VGG	92.5	**89.0**	**92.4**	**91.3**	98.6	**93.8**	**93.8**	**95.4**

Avg.±Std.	VGG16	78.0 ± 5.3	67.2 ± 3.4	92.9 ± 2.3	79.4 ± 2.8	98.4 ± 1.1	90.0 ± 3.1	79.4 ± 2.7	89.3 ± 1.4
	SPP-VGG	94.8 ± 2.2	84.4 ± 4.9	91.2 ± 3.1	90.1 ± 2.3	97.7 ± 0.1	94.3 ± 2.0	91.6 ± 2.5	94.5 ± 1.2
	MSP-VGG	95.9 ± 2.3	87.6 ± 3.6	92.8 ± 2.0	92.1 ± 1.3	98.6 ± 0.5	95.0 ± 0.9	93.3 ± 2.0	95.6 ± 0.5

SPP-VGG and MSP-VGG are short for SPP-based VGGNet and MSP-based VGGNet, respectively. The best results are highlighted in bold. The listed metrics were obtained on the test dataset.

**Table 4:** Precision and F1-score comparisons among VGG16, SPP-based VGGNet, and MSP-based VGGNet.

Fold	Methods	Performance evaluation (%)							
		PRE_ER_	PRE_IM_	PRE_EL_	$\bar{\text{PRE}}$	F1‐score_ER_	F1‐score_IM_	F1‐score_EL_	$\bar{\text{F}1‐\text{score}}$
1	VGG16	89.1	82.5	83.3	85.0	85.7	77.7	87.7	83.9
	SPP-VGG	93.0	84.5	93.7	90.4	94.3	87.7	90.4	90.8
	MSP-VGG	**94.4**	**88.2**	**93.8**	**92.1**	**96.5**	**89.6**	**91.7**	**92.6**

2	VGG16	93.2	73.2	86.0	84.2	88.7	70.3	89.2	82.9
	SPP-VGG	92.8	**89.3**	94.7	92.3	95.5	88.2	94.0	92.6
	MSP-VGG	**94.1**	88.6	**95.9**	**92.9**	**96.2**	**89.7**	**94.3**	**93.5**

3	VGG16	96.2	69.2	81.6	82.4	81.6	67.9	87.50	79.7
	SPP-VGG	94.3	80.5	86.4	87.1	93.0	78.5	88.2	86.5
	MSP-VGG	**98.6**	**86.3**	**90.4**	**91.7**	**96.5**	**85.7**	**91.6**	**91.3**

4	VGG16	**96.3**	76.9	82.9	85.4	86.7	70.4	89.0	82.6
	SPP-VGG	92.5	**91.3**	91.8	91.9	93.2	**86.3**	93.9	91.1
	MSP-VGG	95.5	88.7	**92.4**	**92.2**	**95.5**	85.1	**94.2**	**91.6**

5	VGG16	**98.0**	61.9	80.6	80.2	83.8	62.7	84.6	77.6
	SPP-VGG	92.7	82.4	91.5	88.8	93.3	83.8	90.2	89.1
	MSP-VGG	95.4	**84.9**	**93.7**	**91.3**	**93.9**	**86.9**	**93.1**	**91.3**

Avg.±Std.	VGG16	94.6 ± 3.2	72.8 ± 7.0	82.9 ± 1.8	83.4 ± 1.9	85.5 ± 2.4	69.9 ± 4.8	87.6 ± 1.7	81.3 ± 2.3
	SPP-VGG	93.0 ± 0.6	85.6 ± 4.1	91.6 ± 3.7	90.1 ± 2.0	93.9 ± 0.9	85.0 ± 3.5	91.4 ± 2.2	90.1 ± 2.0
	MSP-VGG	95.6 ± 1.6	87.3 ± 1.5	93.2 ± 1.8	92.0 ± 0.5	95.7 ± 0.9	87.5 ± 1.9	93.0 ± 1.2	92.1 ± 0.8

SPP-VGG and MSP-VGG are short for SPP-based VGGNet and MSP-based VGGNet, respectively. The best results are highlighted in bold. The listed metrics were obtained on the test dataset.

**Table 5:** Training and testing time comparisons among VGG16, SPP-based VGGNet, and MSP-based VGGNet.

Methods	Single time			5-fold time		
	Training	Testing	Total	Training	Testing	Total
VGG16	9 m 42 s	2 m 37 s	12 m 19 s	48 m 30 s	12 m 36 s	61 m 6 s
SPP-based VGGNet	7 m 30 s	35 s	8 m 5 s	37 m 28 s	2 m 44 s	40 m 12 s
MSP-based VGGNet	6 m 54 s	30 s	7 m 24 s	34 m 27 s	2 m 30 s	36 m 57 s

## Data Availability

The data used to support the findings of this study are available from the corresponding author upon request.
